The article "Oral Administration of Electron-Beam Inactivated Rhodococcus equi Failed to Protect Foals against Intrabronchial Infection with Live, Virulent R. equi" was published in 2016. Journal: PLoS One.

# Oral Administration of Electron-Beam Inactivated *Rhodococcus equi* Failed to Protect Foals against Intrabronchial Infection with Live, Virulent *R*. *equi*

**DOI:** 10.1371/journal.pone.0148111

**Published:** 2016-02-01

**Authors:** Joana N. Rocha, Noah D. Cohen, Angela I. Bordin, Courtney N. Brake, Steeve Giguère, Michelle C. Coleman, Robert C. Alaniz, Sara D. Lawhon, Waithaka Mwangi, Suresh D. Pillai

**Affiliations:** 1 Department of Large Animal Clinical Sciences, College of Veterinary Medicine & Biomedical Sciences, Texas A&M University, College Station, Texas, 77843–4475, United States of America; 2 Department of Large Animal Medicine, College of Veterinary Medicine, University of Georgia, Athens, Georgia, 30602–7385, United States of America; 3 Department of Microbial Pathogenesis and Immunology, Texas A&M Health Science Center, College Station, Texas, 77843, United States of America; 4 Department of Veterinary Pathobiology, College of Veterinary Medicine and Biomedical Sciences, Texas A&M University, College Station, Texas, 77843–4467, United States of America; 5 National Center for Electron Beam Research–IAEA Collaborative Centre for Electron Beam Technology, Texas A&M University, College Station, Texas, 77843, United States of America; Institut National de la Santé et de la Recherche Médicale (INSERM), FRANCE

## Abstract

There is currently no licensed vaccine that protects foals against *Rhodococcus equi*–induced pneumonia. Oral administration of live, virulent *R*. *equi* to neonatal foals has been demonstrated to protect against subsequent intrabronchial challenge with virulent *R*. *equi*. Electron beam (eBeam)-inactivated *R*. *equi* are structurally intact and have been demonstrated to be immunogenic when administered orally to neonatal foals. Thus, we investigated whether eBeam inactivated *R*. *equi* could protect foals against developing pneumonia after experimental infection with live, virulent *R*. *equi*. Foals (n = 8) were vaccinated by gavaging with eBeam-inactivated *R*. *equi* at ages 2, 7, and 14 days, or gavaged with equal volume of saline solution (n = 4), and subsequently infected intrabronchially with live, virulent *R*. *equi* at age 21 days. The proportion of vaccinated foals that developed pneumonia following challenge was similar among the vaccinated (7/8; 88%) and unvaccinated foals (3/4; 75%). This vaccination regimen did not appear to be strongly immunogenic in foals. Alternative dosing regimens or routes of administration need further investigation and may prove to be immunogenic and protective.

## Introduction

*Rhodococcus equi* is a Gram-positive, facultative, intracellular pathogen that causes a pyogranulomatous pneumonia in foals approximately 1 to 6 months of age [1, 2]. Virulence of *R*. *equi* in foals is attributable to the presence of an 85- to 90-kilobase (kb) plasmid, including the *vapA* gene which encodes the virulence-associated protein A (VapA) [3–5]. Mature horses are generally not susceptible unless immunocompromised [6, 7]. The reasons for this age-related susceptibility are not fully understood; however, immaturity or naivety of the immune system of foals have been proposed as principal determinants of the outcome of infection [8].

The article "Oral Administration of Electron-Beam Inactivated Rhodococcus equi Failed to Protect Foals against Intrabronchial Infection with Live, Virulent R. equi" was published in 2016. Journal: PLoS One.

Pneumonia induced by *Rhodococcus equi* occurs worldwide, and virulent isolates can be found at horse farms in the air, soil, and feces [9–11]. The disease is problematic for several reasons. First, the insidious progression of *R*. *equi* pneumonia in foals results in marked pathology by the time clinical signs are manifested [12]. Consequently, treatment is generally prolonged, expensive, and not always successful. Screening for earlier detection of disease has been demonstrated to have limited accuracy [13, 14]. Methods for chemo- or immuno-prophylaxis have either been inadequately effective (at best) or unacceptable (e.g., macrolide chemoprophylaxis because of concerns for promoting antimicrobial resistance) [15–18]. Moreover, prophylactic strategies such as transfusion of hyperimmune plasma can be expensive, labor-intensive, and carry some risk for foals [19–23]. Thus, great need exists for an effective vaccine to prevent *R*. *equi* pneumonia in foals.

Currently, no commercial vaccine against *R*. *equi* pneumonia is licensed in the United States, Canada, or European Union. Several vaccines against *R*. *equi* pneumonia have been investigated, including maternal vaccination [24–26], subunit vaccines [27, 28], genetically-modified organisms [29, 30], and DNA vaccines [31–33]. To date, the only method that has been repeatedly documented to protect foals against experimental intrabronchial infection with *R*. *equi* has been oral administration (gavage) of live, virulent *R*. *equi* [34, 35]. While these results are greatly encouraging, the administration of live, virulent organisms as a vaccine is not feasible because of safety concerns for the environment and for foals. Thus, alternative approaches to the use of live, virulent *R*. *equi* should be considered. Recently, our laboratory demonstrated that irradiating live, virulent *R*. *equi* with an electron beam (eBeam) inhibited bacterial replication while maintaining cell wall integrity [36]. Moreover, when administered intragastrically these eBeamed bacteria induced both mucosal and cell-mediated immunity (CMI) [36]. Further studies have shown that eBeam-inactivated bacteria remain metabolically active [37]. Thus, we hypothesized that vaccinating foals with eBeam-inactivated *R*. *equi*, using the same vaccination schedule as was most recently demonstrated to protect foals using orally-administered live, virulent organisms [35], would protect foals against intrabronchial infection with live, virulent *R*. *equi*.

The article "Oral Administration of Electron-Beam Inactivated Rhodococcus equi Failed to Protect Foals against Intrabronchial Infection with Live, Virulent R. equi" was published in 2016. Journal: PLoS One.

## Materials and Methods

### Ethics Statement

All procedures for this study were reviewed and approved by the Texas A&M University Institutional Animal Care and Use Committee (protocol number AUP# IACUC 2013–0171) and the Texas A&M University Institutional Biosafety Committee (permit number 014132-Cohen). The foals used in this study were owned by Texas A&M University, and permission for their use was provided in compliance with the Institutional Animal Care and Use Committee procedures. No foals were euthanized or died during the course of this study.

### Preparation of Bacteria and Electron Beam Irradiation

*Rhodococcus equi* strain EIDL 5–331 (a virulent, *vapA*-gene-positive isolate recovered from a pneumonic foal in Texas) was used for this study. The method for culture and inactivation of *R*. *equi* for vaccine preparation has been described in an earlier publication from our laboratory [36]. Briefly, one colony-forming unit (CFU) was incubated overnight at 37°C in 25 ml of brain-heart infusion (BHI) broth and sub-cultured in 1,000 ml of BHI broth for an incubation of another 24 hr. The bacterial suspension was washed with phosphate-buffered saline (PBS), and resuspended in sterile 0.9% NaCl solution. For eBeam preparation, 25 ml of bacterial suspensions of approximately 1x10^9^ CFU/ml were exposed to a target irradiation dose of 5 kGy using a 10-MeV, 18-kW linear accelerator. Inactivated *R*. *equi* were cultured immediately after irradiation to confirm absence of bacterial replication [36].

### Study Animals

Twelve healthy Quarter Horse foals were used for this study. All foals had age-appropriate results of complete blood count (CBC) on day 2 of life. Individual foals were randomly assigned to a vaccinated group, Group 1 (N = 8), or a control group, Group 2 (N = 4). Group 1 foals received 1 x 10^11^ CFU of *R*. *equi* inactivated by 5 kGy of eBeam irradiation, adjuvanted with 100 μg of the mucosal adjuvant cholera toxin B (CTB, List Biological Laboratories, Campbell, CA, USA), and suspended to a final volume of 100 ml in 0.9% NaCl solution by gavage on days 2, 7, and 14 of life. This dose was previously demonstrated to be immunogenic in foals [36] and represents 10 times the dose of live organisms administered orally in previous studies [34,35]. The frequency of administration was selected to match that used for oral administration of live, virulent *R*. *equi* [35]. Group 2 foals (N = 4) received 100 ml of 0.9% NaCl solution intragastrically at ages 2, 7, and 14 days. The foals in Groups 1 and 2 were housed separately.

The article "Oral Administration of Electron-Beam Inactivated Rhodococcus equi Failed to Protect Foals against Intrabronchial Infection with Live, Virulent R. equi" was published in 2016. Journal: PLoS One.

### Experimental Infection

Foals from Group 1 and 2 were experimentally infected at age 21 days with 1 x 10^6^ CFU of live *R*. *equi* (strain EIDL 5–331, the same strain used for the vaccine). Prior to experimental infection with *R*. *equi*, each foal’s lungs were evaluated by auscultation and thoracic ultrasonography to document absence of pre-existing lung disease. Foals were sedated using intravenous injection of romifidine (0.8 mg/kg; Sedivet, Boehringer-Ingelheim Vetmedica, Inc., St. Joseph, MO, USA) and butorphanol (0.02 mg/kg; Zoetis, Florham Park, New Jersey, USA) to facilitate endoscopy. An aseptically-prepared, videoendoscope with outer diameter of 9-mm was inserted via the nares into the trachea and passed to the bifurcation of the main-stem bronchi. A 40-mL suspension of virulent EIDL 5–331 *R*. *equi* containing approximately 1 x 10^6^ viable bacteria was administered transendoscopically, with 20 ml infused into the right mainstem bronchus and 20 ml into the left mainstem bronchus. The channel was flushed twice with 20 ml of air after each 10 ml bacterial infusion.

### Sample Collection

Blood samples were collected from foals and their dams on day 2 (prior to vaccination), on day 21 (post-vaccination, pre-challenge), and day 84 (post-challenge) of foals’ age. A total of 43 ml of blood was collected from each foal from a jugular vein into Vacutainer^TM^ tubes: 16 ml of blood was collected into 2 tubes without anticoagulant and centrifuged at 3,000 x g for 5 min to harvest serum, which was separated and frozen at -80°C until assayed; 24 ml of blood was collected into 3 tubes with sodium heparin as an anticoagulant for isolation of peripheral blood mononuclear cells (PBMCs); and, 3 ml of blood was collected into a tube with 5.4 mg EDTA as an anticoagulant to perform a CBC. A total of 24 ml of blood was collected from each mare from a jugular vein into 3 Vacutainer^TM^ tubes with sodium heparin as anticoagulant for isolation of peripheral blood mononuclear cells (PBMCs). Naso-pharyngeal samples were collected from foals on days 2, 21, and 84 by inserting a 26-mm white plastic foam plug (Identi-Plug, Jaece Industries Inc, North Tonawanda, NY, USA), introduced with an equine insemination pipet, to the nasal ventral meatus. The foam plug was left in the nasal cavity for 5 min, and the naso-pharyngeal liquid was collected by centrifugation in a 50-ml conical tube at 500 x g for 10 min and frozen at -80°C until assayed. Transendoscopic tracheobronchial aspirate (T-TBA) fluid was collected 3 times from foals in both groups: on day 21 (pre-challenge); at the time of clinical diagnosis with *R*. *equi* pneumonia; and, either when clinical signs of *R*. *equi* pneumonia ceased to exist or at age 84 days (i.e., end of study) if foals remained healthy. The T-TBAs were performed using a 1-meter endoscope which was disinfected with glutaraldehyde, and then rinsed with 1 X PBS prior to the procedure. The T-TBA was obtained by sedating foals with romifidine (0.8 mg/kg; Sedivet, Boehringer-Ingelheim Vetmedica, Inc., St. Joseph, MO, USA) and washing the tracheobronchial tree with 0.9% NaCl solution delivered through a triple-lumen, double-guarded sterile tubing system (MILA International, Inc, Erlanger, KY, USA).

The article "Oral Administration of Electron-Beam Inactivated Rhodococcus equi Failed to Protect Foals against Intrabronchial Infection with Live, Virulent R. equi" was published in 2016. Journal: PLoS One.

### Foal Monitoring and Diagnostic Criteria

Beginning with the day of infection, rectal temperature, heart rate, and respiratory rate of the foals were monitored and recorded twice daily. Clinical signs of abnormal lung sounds, coughing, lethargy, respiratory effort, nasal discharge, and polysynovitis also were monitored and recorded twice daily. The lungs were monitored weekly using thoracic ultrasonography for evidence of peripheral pulmonary consolidation or abscess formation.

Foals were considered to manifest clinical signs of pneumonia when they had ultrasonographic evidence of pulmonary abscessation or consolidation with maximal lesion diameter ˃ 2.0 cm and either a rectal temperature of ˃ 39.7°C, a cough at rest, or both fever (˃ 39.7°C) and cough. On the day a foal was diagnosed with pneumonia, a CBC, thoracic ultrasonography, and T-TBA were performed. The T-TBA fluid was submitted to the Texas Veterinary Medical Diagnostic Laboratory, College Station, for cytologic examination and for microbiologic culture. Foals were considered to have a diagnosis of *R*. *equi* pneumonia if they met the aforementioned criteria for clinical signs of pneumonia and had cytologic evidence of septic inflammation with Gram-positive pleomorphic rods and *R*. *equi* recovered by microbiologic culture of T-TBA fluid. Foals were monitored through 84 days of age. Foals that did not have clinical signs of disease, but had ultra-sonographic evidence of lung lesions, were monitored through 84 days of age.

### Treatment of Study Foals

Foals diagnosed with *R*. *equi* pneumonia were treated with either the combination of clarithromycin (7.5 mg/kg; PO; q 12 hr) and rifampin (5 mg/kg; PO, q 12 hr) or liposomal gentamicin solution (6.6 mg/kg, q 24 hr) [38] diluted in 250 ml of 0.9% NaCl given via slow intravenous infusion over 15 min. Foals were treated as deemed necessary by attending veterinarians (AIB; NDC; MCC) with flunixin meglumine (0.6 to 1.1 mg/kg; PO) for discomfort and fever. Foals were treated until clinical signs and thoracic ultrasonographic lesions resolved.

The article "Oral Administration of Electron-Beam Inactivated Rhodococcus equi Failed to Protect Foals against Intrabronchial Infection with Live, Virulent R. equi" was published in 2016. Journal: PLoS One.

### Cell-Mediated Immune Response

The CMI response to vaccination was assessed by interferon-γ (IFN-γ) production by peripheral blood mononuclear cells (PBMCs) following specific stimulation with an *R*. *equi* antigen (strain EIDL 5–331). The protocol for preparation of *R*. *equi* antigen has been described previously [39]. The PBMCs were isolated using a Ficoll-Paque gradient separation (GE Healthcare, Piscataway, NJ, USA) and resuspended in 1X RPMI-1640 media with L-glutamine (Gibco, Life Technologies, Grand Island, NY, USA), 15% fetal bovine serum (Gibco, Life Technologies, Grand Island, NY, USA), and 1.5% penicillin-streptomycin (Gibco, Life Technologies, Grand Island, NY, USA). The PBMCs were cultured for 48 h at 37°C with 5% CO_2_ with either media only, the mitogen Concanavalin A (positive control; 2.5 mg/ml, Sigma-Aldrich, St. Louis, MO, USA), or *R*. *equi* antigen representing multiplicity of infection of 10. After 48 h, supernatants from each group were harvested and frozen at -80°C until examined for IFN-γ production using an equine IFN-γ enzyme linked immunosorbent assay (ELISA) kit (Mabtech AB, Nacka Strand, Stockholm, Sweden) according to manufacturer’s instructions. Optical densities (OD) were determined using a microplate reader Synergy 2 (Biotek, Winooski, VT, USA); standard curves were generated and IFN-γ concentrations in each sample were calculated for each isotype using the software Gen 5 (Biotek, Winooski, VT, USA). Mare PBMCs were tested along with each sample from their foals as controls to ensure that positive (i.e., Concanavilin A) and negative (i.e., media only) stimuli were functioning as expected because we anticipated that PBMCs of younger foals might be less responsive to ConA stimulation.

### Mucosal and Systemic Humoral Immune Responses

Mucosal humoral immune responses were assessed by quantifying *R*. *equi*-specific IgA in naso-pharyngeal eluates. Systemic humoral response was assessed among foals by quantifying serum concentrations of *R*. *equi*-specific IgA and IgG sub-isotypes. Concentrations *R*. *equi*-specific IgA and IgG sub-isotypes were determined by ELISA as previously described [36]. Briefly, ELISA plates (Maxisorp, Nalge Nunc International, Rochester, NY) were coated with 2.5 mg/ml of *R*. *equi* antigen (same *R*. *equi* antigen as mentioned above) diluted in coating buffer (Carbonate-bicarbonate buffer, Sigma-Aldrich, St. Louis, MO) overnight at 4°C. Plates were washed 5 times with Tris buffered saline (TBS) with 0.005% Tween 20, blocked with 200 ml TBS with 1% BSA for 30 min at room temperature (RT), and washed again. Serum samples (diluted 1:32) from study foals, a positive control of *R*. *equi* hyperimmune plasma (Mg Biologics, Ames, IA) diluted at concentrations of 1:40, 1:320, 1:10, and 1:320 for IgGa, IgGb, IgG(T), and IgA, respectively, and a negative control of undiluted fetal horse serum (Biowest, Miami, FL, USA) were added in duplicates to the wells. Naso-pharyngeal (NP) swab eluates were assayed undiluted. After another washing, goat anti-horse IgA (Bethyl Laboratories, Montgomery, TX, USA), IgGb (Lifespan Biosciences, Seattle, WA), or IgG(T) (Bethyl Laboratories, Montgomery, TX, USA) peroxidase conjugated, or mouse anti-horse IgGa peroxidase conjugated (AbD Serotec, Raleigh, NC, USA) were added to the wells and incubated for 60 min at RT. Plates were washed again, and TMB One Component HRP Microwell Substrate (Bethyl Laboratories, Montgomery, TX) was added to the wells and incubated for 15 min at 22°C in the dark. The reaction was stopped by adding sulfuric acid solution to the wells. Optical densities were determined by using microplate reader Synergy 2 (Biotek, Winooski, VT, USA).

The article "Oral Administration of Electron-Beam Inactivated Rhodococcus equi Failed to Protect Foals against Intrabronchial Infection with Live, Virulent R. equi" was published in 2016. Journal: PLoS One.

### Data Analysis

#### Clinical data

Data were analyzed using descriptive and inferential methods. For descriptive purposes, categorical data were summarized in contingency tables and continuous data were summarized as medians and ranges. Categorical data were compared using Fisher’s exact tests and continuous variables were compared using a Wilcoxon rank-sum test.

#### CMI data (IFN-γ expression by cultured PBMCs)

Data were analyzed using linear mixed-effects (LME) models to account for repeated measures on foals. The outcome variable was IFN-γ expression, which was transformed using the function log_10_ (concentration + 1); the addition of 1 was necessary because there were values of 0 for some foals at some times.

#### Serum and nasal antibody concentration data

The optical density (OD) values for a given foal at a given age were divided by the plate positive control value to account for plate-to-plate variation; each foal’s serum samples from all 3 time-points were tested on a single plate (i.e., the same plate). Data were analyzed using linear mixed-effects modeling. The outcome (dependent) variable was the relative OD (i.e., sample OD/positive control); age, vaccine group, and their interaction terms (i.e., age x group) were modeled as fixed, categorical effects, and foal was modeled as a random effect to account for repeated measures. Model fit was assessed graphically using diagnostic residual plots. When model fit appeared poor, data were transformed (log_10_) to improve fit, and model fit was again assessed using diagnostic residual plots.

The article "Oral Administration of Electron-Beam Inactivated Rhodococcus equi Failed to Protect Foals against Intrabronchial Infection with Live, Virulent R. equi" was published in 2016. Journal: PLoS One.

## Results

### Clinical Outcomes

All foals developed lesions ≥ 2 cm in their peripheral lungs identified by thoracic ultrasonography. The primary study outcome was the proportion of foals that developed clinical signs of pneumonia as defined above. Ten of 12 infected foals (83%) developed clinical signs of pneumonia, and isolation of virulent *R*. *equi* and cytologic evidence of sepsis was observed for the TBA fluid of all foals at the time clinical signs of pneumonia were observed. There was no significant (P = 0.9999; Fisher’s exact test) difference in the proportion of foals that developed clinical signs of pneumonia among the control foals (75%; 3/4) and the vaccinated foals (88%; 7/8). All affected foals had fever, cough, abnormal lung sounds or tracheal rattle, and ultrasonographic evidence of pulmonary consolidations. There were no significant differences in foals in the age at onset of clinical signs, duration of clinical signs, or lesion sizes (Tables 1 and 2. Of the study foals, 1 of the 4 control foals (25%) and 4 of the 8 vaccinated foals (50%) developed polysynovitis associated with experimental *R*. *equi* pneumonia; there was no significant difference in these proportions (P = 0.5758; Fisher’s exact test).

**Table 1:** Ages at onset of clinical signs and ultrasonographic lesions of vaccinated and control foals. There were no significant differences between the two groups.

Variable	Controls (N = 4) Median (Range)	Vaccinates (N = 8) Median (Range)	P^#^
Age at onset of coughing (days)	34 (26 to 39)	43 (27 to 37)	0.7758
	N = 4	N = 7	
Age at onset of tachypnea* (days)	21.5 (20 to 27)	23.5 (21 to 35)	0.3031
	N = 4	N = 8	
Age at onset of fever (days)	34 (30 to 37)	36 (33 to 42)	0.9076
	N = 3	N = 7	
Age at onset of ultrasound lesions (days)	36.5 (34 to 39)	37 (33 to 46)	0.9999
	N = 4	N = 8	
Age of maximal diameter of ultrasound lesions (days)	39.5 (36 to 49)	42 (33 to 54)	0.8649
	N = 4	N = 8	

^#^ P values from Wilcoxon rank-sum test

* Tachypnea defined as respiratory rate > 60

**Table 2:** Duration of clinical signs and ultrasonographic lesions of vaccinated and control foals. There were no significant differences between the 2 groups.

Variable	Controls (N = 4) Median (Range)	Vaccinated (N = 8) Median (Range)	P^#^
Duration of coughing (days)	7.5 (4 to 19)	13 (4 to 24)	0.2964
	N = 4	N = 7	
Duration of tachypnea* (days)	36.5 (27 to 57)	33.5 (15 to 59)	0.7972
	N = 4	N = 7	
Duration of fever (days)	2 (1 to 13)	5 (1 to 17)	0.9079
	N = 3	N = 7	
Duration of fever (days) including the foal that had 0 days	1.5 (0 to 13)	3.5 (0 to 17)	0.6678
	N = 3	N = 8	
Duration of ultrasound lesions (days)	21 (7 to 42)	17.5 (7 to 43)	0.9999
	N = 4	N = 8	
Duration of abnormal lung sounds (days)	5.5 (1 to 29)	25 (2 to 34)	0.2183
	N = 4	N = 7	
Duration of abnormal lung sounds (days) including the foal that had 0 days.	5.5 (1 to 29)	21.5 (0 to 34)	0.4439
	N = 4	N = 8	
Duration of depressed attitude (days)	4.5 (0 to 16)	11 (0 to 33)	0.2654
	N = 4	N = 8	
Duration of antimicrobial treatment (days)	35 (13 to 41)	25 (12 to 42)	0.5676
	N = 3	N = 7	
Duration of antimicrobial treatment (days) including the foal that had 0 days	24 (0 to 41)	24.5 (0 to 42)	0.9321
	N = 4	N = 8	
Duration of diarrhea (days)	3 (1 to 8)	3 (2 to 8)	0.8778
	N = 3	N = 5	

^#^ P values from Wilcoxon rank-sum test

* Tachypnea defined as respiratory rate > 40

The article "Oral Administration of Electron-Beam Inactivated Rhodococcus equi Failed to Protect Foals against Intrabronchial Infection with Live, Virulent R. equi" was published in 2016. Journal: PLoS One.

### Serum and Nasal *R*. *equi*-Specific Antibody Responses

#### Serum IgGa

There was no significant effect of either vaccination or the interaction of vaccination and time (i.e., no modification of effects of time by vaccination group; Fig 1) on serum concentrations of anti-*R*. *equi*-specific IgGa. For these data, log_10_ transformation was deemed appropriate for analysis to ensure good model fit. Concentrations of IgGa were significantly (P = 0.0120; LME) lower for foals in both groups at age 21 days (controls: mean relative OD = 0.19; 95% confidence interval = 0.11 to 0.29; vaccinates: mean relative OD = 0.11; 95% confidence interval = 0.07 to 0.19), than at age 2 days (controls: mean relative OD = 0.34; 95% confidence interval = 0.20 to 0.57; vaccinates: mean relative OD = 0.20; 95% confidence interval = 0.11 to 0.36). Concentrations of *R*. *equi*-specific IgGa at day 84 were not significantly greater than baseline, although it appeared that IgGa values were higher than baseline for the eBeam vaccinated foals (Fig 1). Concentrations of IgGa were significantly (P < 0.05; LME) greater at age 84 days than age 21 days for foals in both groups (controls: mean relative OD = 0.62; 95% CI = 0.40 to 0.97; vaccinates: mean relative OD = 0.37; 95% CI = 0.24 to 0.58).

**Fig 1:** Relative OD of IgGa against *R*. *equi* in control foals (left panel labeled C) and vaccinated foals (right panel labeled V). Both groups tended to decrease between days 2 and 21, but this difference was not significant; however, both groups increased significantly between days 21 and 84.

#### Serum *R*. *equi*-specific IgGb

There was no significant effect of either vaccination or the interaction of vaccination and time (i.e., no modification of effects of time by vaccination group; Fig 2) on serum concentrations of IgGb. Concentrations of IgGb were, however, significantly (P = 0.0003; LME) lower for foals in both groups at age 21 days (controls: mean relative OD = 0.25; 95% confidence interval = 0.16 to 0.34; vaccinates: mean relative OD = 0.21; 95% confidence interval = 0.12 to 0.30), than at age 2 day (controls: mean relative OD = 0.44; 95% confidence interval = 0.26 to 0.63; vaccinates: mean relative OD = 0.40; 95% confidence interval = 0.21 to 0.58). Although values for both groups appeared (Fig 2) to be lower at day 84 than day 2, this difference was not significant. Although OD values tended to increase from day 21 to day 84, this difference also was not significant.

The article "Oral Administration of Electron-Beam Inactivated Rhodococcus equi Failed to Protect Foals against Intrabronchial Infection with Live, Virulent R. equi" was published in 2016. Journal: PLoS One.

**Fig 2:** Relative OD of IgGb against *R*. *equi* in control foals (left panel labelled C) and vaccinated foals (right panel labelled V). Both groups decreased significantly between days 2 and 21; although values tended to be lower at day 84, this difference was not significant.

#### Serum *R*. *equi*-specific IgG(T)

There was no significant effect of either vaccination or the interaction of vaccination and time (i.e., no modification of effects of time by vaccination group; Fig 3) on serum concentration of IgG(T). Concentrations of IgG(T) were, however, significantly (P = 0.0230; LME) lower for foals in both groups at age 21 days (controls: mean relative OD = 0.31; 95% confidence interval = 0.15 to 0.47; vaccinates: mean relative OD = 0.17; 95% confidence interval = 0.01 to 0.33), than at age 2 days (controls: mean relative OD = 0.50; 95% confidence interval = 0.26 to 0.73; vaccinates: mean relative OD = 0.36; 95% confidence interval = 0.07 to 0.64). Values for both groups at day 84 (controls: 0.96; 95% CI = 0.81 to 1.12; vaccinates: 0.82; 95% CI = 0.66 to 0.98) were significantly (P < 0.05; LME) different than values for foals in that group at ages 2 or 21 days.

**Fig 3:** Relative OD of IgG(T) against *R*. *equi* in control foals (left panel labelled C) and vaccinated foals (right panel labelled V). Both groups decreased significantly between days 2 and 21; values at day 84 were significantly greater than those at either day 2 or 21.

#### Serum *R*. *equi*-specific IgA

There was no significant effect of either vaccination or the interaction of vaccination and time (i.e., no modification of effects of time by vaccination group) on serum concentration of IgA. Although concentrations of IgA were higher for foals in both groups at age 21 days (controls: mean relative OD = 0.69; 95% confidence interval = 0.34 to 1.04; vaccinates: mean relative OD = 0.80; 95% confidence interval = 0.45 to 1.15), than at age 2 days (controls: mean relative OD = 0.39; 95% confidence interval = 0.03 to 0.76; vaccinates: mean relative OD = 0.51; 95% confidence interval = 0.15 to 0.88), the difference was not significant. Values for both groups at day 84 were similar to age 2 days (controls: mean relative OD = 0.42; 95% confidence interval = 0.07 to 0.77; vaccinates: mean relative OD = 0.54; 95% confidence interval = 0.18 to 0.91) and not significantly different than values for foals in that group at age 21 days.

The article "Oral Administration of Electron-Beam Inactivated Rhodococcus equi Failed to Protect Foals against Intrabronchial Infection with Live, Virulent R. equi" was published in 2016. Journal: PLoS One.

#### Nasal *R*. *equi-*specific IgA

Although values of the relative OD (Fig 4) tended to increase at day 21 for several foals, there were no significant effects of time, group, or their interaction on nasal IgA values.

**Fig 4:** Relative OD of IgA against *R*. *equi* in control foals (left panel labelled C) and vaccinated foals (right panel labelled V). There were no significant effects of time or group.

### CMI Responses

Stimulation with ConA resulted in significant (P < 0.0001; LME) induction of IFN-γ expression by PBMCs of foals at all ages (Fig 5). Responses to ConA were significantly greater on day 21 (P = 0.0060; LME) and on day 84 (P = 0.0160; LME) than on day 2; however the responses to ConA did not differ between foals at day 21 and day 84. Basal expression of INF-γ did not change among ages (Fig 5). Although *R*. *equi* antigen did not stimulate a significant increase in IFN-γ expression on day 2, responses on day 21 and day 84 were significantly (P < 0.0001; LME) greater than those observed on day 2 (Fig 5). Moreover, the magnitude of expression of IFN-γ on day 84 was significantly (P = 0.0196; LME) greater than that of day 21 (Fig 5).

**Fig 5:** Production of IFN-γ by PBMCs exposed to stimuli at ages 2, 21, and 84 days in 12 foals. Circles represent unvaccinated foals (N = 4) and triangles represent vaccinated foals (N = 8). The mitogen (concavalin A) induced significantly (P < 0.0001; LME) greater expression of IFN-γ relative to the unstimulated PBMCs (Control) at each age; moreover, expression induced at days 21 and 84 was significantly (P = 0.0060 and 0.0160, respectively; LME) greater than that induced on day 2. There was no significant difference among ages for the unstimulated control samples. Stimulation with *R*. *equi* did not induce expression of IFN-γ relative to unstimulated control cells on day 2, but did induce significant expression on days 21 and 84 (P < 0.0001; LME) relative to baseline, and expression was significantly greater (0.0196; LME) on day 84 (following infection) than 21 (prior to infection).

Our primary objective for CMI testing was to compare IFN-γ production by stimulated PBMCs by age between vaccinated and unvaccinated foals. For a given age, there was no significant effect of vaccination on IFN-γ production (Fig 6). Significant effects of age, however, were observed: stimulation with *R*. *equi* antigen generated significantly (P < 0.0001; LME) greater IFN-γ production at ages 21 and 84 days relative to day 2, and responses on day 84 were significantly (P < 0.0095; LME) greater on day 84 than on day 21. Graphically, it appeared that there was an outlier among control foals at age 21 days and evaluation of diagnostic residual plots indicated this observation was highly influential. When this observation was excluded, significant effects of age, vaccination, and their interaction were observed. Excluding this foal, the IFN-γ responses were significantly greater at age 21 days (P < 0.05; LME) for the vaccinated foals than the controls, but there was no significant difference between groups at either age 2 days (prior to vaccination) or age 84 days (after intrabronchial infection). Among the control foals, IFN-γ expression in response to treatment was significantly (P < 0.05; LME) greater on day 84 than either days 2 or 21, but values on days 2 and 21 were not significantly different. Among the vaccinated foals, values of IFN-γ were significantly (P < 0.05; LME) greater at day 21 and 84 than day 2, but did not differ significantly between days 21 and 84. These data indicate that, when the outlier was excluded, CMI was significantly (P < 0.05; LME) greater in the vaccinated foals than control foals on day 21 (prior to infection). Interestingly, the foal with the outlier observation was the control foal that did not develop clinical signs of pneumonia following infection.

The article "Oral Administration of Electron-Beam Inactivated Rhodococcus equi Failed to Protect Foals against Intrabronchial Infection with Live, Virulent R. equi" was published in 2016. Journal: PLoS One.

**Fig 6:** Production of IFN-γ by PBMCs exposed to *R*. *equi* antigen at ages 2, 21, and 84 days in 12 foals: 4 control foals that were unvaccinated and 8 foals vaccinated intragastrically with an eBeam vaccine. No significant effect of vaccine was observed, but concentrations of IFN-γ increased significantly (P < 0.0001; LME) at ages 21 and 84 days relative to controls, and values were significantly higher on day 84 than 21. A value for 1 control foal on day 21 was considered to be an outlier (arrow). When this value was excluded, significant effects of vaccination that varied by age were observed: excluding this value, the vaccinated group had significantly (P < 0.05; LME) higher IFN-γ expression than control foals on day 21 (but not at the other ages; see text for details).

## Discussion

The eBeam-inactivated *R*. *equi* vaccine was not effective in protecting foals against experimental infection with live virulent *R*. *equi*. *Ten* of the 12 foals became clinically affected with pneumonia, and there was no significant difference in the proportion developing pneumonia among the vaccinated foals (88%; 7/8) or the control foals (75%; 3/4). Furthermore, clinical parameters such as age at onset or duration of cough, fever, abnormal lung sounds, and ultrasonographic lesions did not differ significantly between groups. Only age at onset of tachypnea differed significantly between groups. In light of other findings, we consider this finding to be the result of chance. It should be noted that all foals in all groups developed at least 1 thoracic ultrasonographic lesion > 1 cm in diameter (including the 2 foals that remained free of clinical pneumonia). In the clinical experience of the authors, the observed clinical signs and thoracic ultrasonographic lesions were similar to those observed with naturally-occurring *R*. *equi* pneumonia in foals. As observed with other relatively low-dose challenge models [40,41], not all foals developed clinical signs following intrabronchial infection. This is consistent with observations that many foals naturally infected may develop sub-clinical infection [40,42,43].

The article "Oral Administration of Electron-Beam Inactivated Rhodococcus equi Failed to Protect Foals against Intrabronchial Infection with Live, Virulent R. equi" was published in 2016. Journal: PLoS One.

The eBeam vaccine did not elicit either systemic humoral or mucosal humoral immune responses. A previous report from our laboratory similarly documented that oral administration of eBeamed virulent *R*. *equi* failed to elicit systemic humoral immune responses [36]; however, in that study there was evidence that vaccination stimulated a significant increase in nasal IgA against *R*. *equi*. Reasons for this discrepancy in IgA responses between these studies are unknown. One possibility is that the previous study used 4 intragastric vaccinations during the first 21 days of age, whereas in this study we performed only 3 intragastric vaccinations during the first 14 days of age. Conceivably, the responses observed in our previous report might have resulted from the additional vaccine dose. Alternatively, foals might have developed stronger and thus detectable responses at an older age (i.e., at 30 days as in the previous study rather than at age 21 days as for this study). Our rationale for decreasing from 4 to 3 doses of vaccine for this study were to mimic the design of the most recent report documenting the efficacy of oral administration of live *R*. *equi* to protect against challenge at 21 days of age [35], to evaluate responses to challenge earlier in life than 30 days, and because our belief that giving fewer vaccines would be associated with better adaptation and compliance by veterinarians and farm staff.

All serum sub-isotypes of IgG (i.e., IgGa, IgGb, and IgG(T)) decreased from day 2 to day 21 in foals of both groups. This decrease was attributed to decay of maternal transfer of antibodies [44]. Values of serum *R*. *equi-*specific IgGa increased from day 21 (pre-infection) to day 84 (post-infection), indicating that serum IgGa might be a marker of infection; however, the values for age 84 weren’t significantly greater than those for day 2, indicating that this response was neither very robust nor consistent. Serum concentrations of IgGb did not appear to increase following infection and thus appeared to be a poor indicator of exposure and disease. In contrast, IgG(T) increased significantly between day 21 and 84 and the values at day 84 were also significantly greater than those at day 2. These results using a whole-cell *R*. *equi* antigen are consistent with a recent report indicating that IgGb specific for VapA was not useful either for diagnosis or prediction (screening) in foals with naturally-occurring or experimental pulmonary infection with *R*. *equi* [45], but that VapA-specific IgGa and IgG(T) were significantly increased following maternal decay, and that the magnitude of increase was greater for IgG(T) [46, 47]. IgGa is thought to be induced by a Th1-biased immune response, which is vital for intracellular pathogenic elimination, whereas IgGb and IgG(T) are thought to result from a Th2-type immune response [48]. Because Th1-type immune responses are considered to be important for control of intracellular pathogens, it has been suggested that those foals that develop *R*. *equi* pneumonia are biased towards an ineffective Th2-type response [48]. Alternatively, progression of the disease process might result in sub-isotype class switching. High titers of IgG(T) are important as they opsonize *R*. *equi* and engage the Fc receptors in neutrophils, which have decreased phagocytic and killing capacities in the neonatal foal [49–51]. This engagement of IgG(T) to the Fc receptors increases phagocytosis of *R*. *equi* by opsonization [46]. As noted previously [47], further evaluation of IgG(T) for diagnostic and screening purposes is warranted.

The article "Oral Administration of Electron-Beam Inactivated Rhodococcus equi Failed to Protect Foals against Intrabronchial Infection with Live, Virulent R. equi" was published in 2016. Journal: PLoS One.

A significant CMI response to the *R*. *equi* strain used for the vaccine as measured by IFN-γ expression by cultured PBMCs was observed when an influential statistical outlier was excluded: IFN-γ responses were not significantly different on day 2 (prior to vaccination) for both control and vaccinated foals, but by day 21 vaccinated foals showed a significantly greater IFN-γ response than the controls. At age 84 days, neither vaccinated nor unvaccinated foals differed in their IFN-γ production. These findings are consistent with our previous results documenting evidence of intragastric vaccination of eBeamed *R*. *equi* eliciting CMI responses. Our latest CMI results must be interpreted with caution because statistical significance was only observed when an outlier was excluded, and this outlier was a control (unvaccinated foal) with a very high CMI response. Interestingly, this control foal was the 1 control foal that did not develop clinical pneumonia following challenge. Regardless, the CMI responses observed in this study in response to vaccination were not protective against intrabronchial infection. As expected, we observed increased production of IFN-γ with age in response to either stimulus (the mitogen ConA [positive control] or the *R*. *equi* antigen). Foals express less IFN-γ early in life [52–54]. This inability to express IFN-γ likely impairs the ability of young foals to mount a robust Th1-based cell mediated immune response, thereby contributing to their susceptibility to intracellular pathogens such as *R*. *equi*. This might also contribute to inefficient antigen priming that impairs the foal’s ability to respond to antigens [55, 56].

There are a number of reasons why this vaccine might have failed in this study to protect foals despite previous evidence of immunogenicity. Whereas live organisms multiply, the eBeam inactivated bacterial cells do not: thus, it is possible that the magnitude of the antigenic load delivered to the gastrointestinal tract might have been inadequate to stimulate immune responses that protected against infectious challenge. Conceivably, a larger dose or more frequent administration of intragastric eBeamed *R*. *equi* might have provided protection. In our previous study of the immunogenicity of oral, virulent *R*. *equi* in foals, we used a similar dose of vaccine but administered 4 doses rather than the 3 doses administered for this project [36]. Alternatively, some degree of intracellular replication might be required to stimulate protective immunity. It is also possible that the route of vaccine administration may not have been optimal.

Although it is generally considered that CMI responses are essential for immunity to intracellular pathogens, evidence exists that humoral systemic immune responses can provide protection. In our previous study [36] we noted that oral administration of live, virulent *R*. *equi* stimulated a systemic *R*. *equi*-specific IgGa response whereas the oral eBeam vaccine did not. Conceivably, antibody responses might be essential for protection against *R*. *equi*. Evidence exists that transfusion of hyperimmune plasma can protect foals against experimentally-induced and naturally-occurring *R*. *equi* pneumonia,[19–23] although conflicting evidence exists [23, 57].

In summary, our eBeam-inactivated vaccine was neither strongly immunogenic nor protective against experimental infection with live, virulent *R*. *equi*. Despite these initial disappointing results, this type of vaccine approach should not be entirely dismissed because a higher dose, stronger dose, more frequent administration, or an alternative method of administration needs to be evaluated. Further understanding of the mechanisms that provide protection to foals when administered live, virulent *R*. *equi* and availability of a small animal model of *R*. *equi* pneumonia would further facilitate vaccine development.
